This article has been retracted.

# Effect of Baogong Zhixue Granules Combined with Tranexamic Acid Injection on the Hemodynamics and Reproductive System in Patients with Postpartum Hemorrhage after Cesarean Section

**DOI:** 10.1155/2022/1249779

**Published:** 2022-06-09

**Authors:** Xuena Cui, Yuzhi Ji, Lijuan Zhang, Qiulan Lv, Ling Liu

**Affiliations:** Department of Obstetrics, The Affiliated Hospital of Qingdao University, Qingdao, 266003, Shandong, China

## Abstract

**Objective:**

To investigate the effect of Baogong Zhixue granules combined with tranexamic acid injection on the hemodynamics and reproductive system in patients with postpartum hemorrhage (PPH) after cesarean section.

**Methods:**

The data of 90 puerperae undergoing cesarean section in our hospital from January 2019 to January 2020 were retrospectively analyzed. According to the order of admission, they were equally divided into the control group (CG) and experimental group (EG). CG was treated with tranexamic acid injection combined with oxytocin, while EG was treated with Baogong Zhixue granules combined with tranexamic acid injection to compare the clinical observation indexes between the two groups.

**Results:**

Compared with CG, EG achieved remarkably less amount of bleeding at 2 h and 24 h after delivery (*P* < 0.001), lower postpartum APTT, PT, HR, and MAP (*P* < 0.001), shorter maintenance time of uterine contraction and lochia (*P* < 0.001), and lower postpartum FSH and LH (*P* < 0.001). After delivery, EG had higher postpartum Fib and descending speed of uterine fundus and *E*_2_ compared with CG (*P* < 0.001).

**Conclusion:**

Baogong Zhixue granules combined with tranexamic acid injection have little effect on the reproductive system of PPH patients after cesarean section, stabilize the hemodynamics, and improve the coagulation function. Therefore, further research on the combined treatment can provide better hemostatic schemes for such patients.

## 1. Introduction

In recent years, the family-planning policy has been constantly adjusted in China. According to relevant literature, the two-child policy was implemented in families with both parents from one-child family and families with a parent from one-child family successively from 2011 to 2013 and was open for all families in 2015. Until 2021, an overall three-child policy in China results in an increasing number of women in need of fertility [1–3]. With the popularization of fertility policy, delivery modes have gradually become a hot topic [4, 5]. Delivery modes are divided into cesarean section and vaginal delivery, and different modes are closely related to the prognosis and health of mothers and infants. Most pregnant women can complete natural vaginal delivery after full-term pregnancy, while a few women are not fit for this mode due to abnormal birth canal and insufficient fertility, and clinicians will perform cesarean section to terminate pregnancy [6, 7]. Cesarean section, as a common midwifery operation in obstetrics and gynecology, is an effective means to save the lives of mothers and infants. However, relevant literature has pointed out that 70% of maternal deaths worldwide are caused by direct obstetric factors and the rest are caused by indirect factors. Among the factors, the main one leading to maternal deaths worldwide is bleeding, and more than 2/3 of the reported deaths from bleeding result from postpartum hemorrhage [8, 9]. Meanwhile, uterine contraction fatigue, retention of placenta, soft obstetrical canal crack, and coagulopathy are the main incentives of postpartum hemorrhage (PPH). In clinics, postpartum hemorrhage refers to the amount of bleeding over 500 ml in puerperae with vaginal delivery or over >1000 ml in those with cesarean section within 24 hours after the delivery of the fetuses [10]. Since the mortality rate of pregnant women is high in the first 24 hours after delivery, routine prevention and active management are mainly adopted in clinical practice to avoid such problems. If the patients were in serious condition and bleeding cannot be controlled, surgical treatment will be adopted to reduce the PPH amount.

There are many clinical studies on the treatment of PPH, and different treatment methods vary in the hemostatic effect, effect on hemodynamics, and other adverse effects on the body. At present, though oxytocin is the main clinical drug to treat PPH with a good effect and rapid onset, its single use does not meet the expectations for its short half-life, accompanied by adverse reactions such as decreased blood pressure. Therefore, more clinical research studies focus on the combination of drugs to improve the hemostatic effect [11, 12]. Baogong Zhixue granules, a compound prescription with the effects of cooling blood for hemostasis and promoting blood circulation to remove blood stasis, are widely used in obstetrics and gynecology, and the effect has been confirmed in the treatment of diseases after normal childbirth and prolonged menstruation [13]. At the same time, Baogong Zhixue granules are suitable for the functional uterine hemorrhage and uterine hemorrhage after the upper ring, which can effectively control bleeding, promote the endometrial repair and evacuation of the intrauterine residual tissue, and reduce the complications. However, few studies have reported the effect of Baogong Zhixue granules combined with tranexamic acid injection on PPH patients after cesarean section. Therefore, this study adopted the combined regime to analyze its application value by observing its effect on the hemodynamics and reproductive system of patients after treatment.

## 2. Materials and Methods

### 2.1. General Information

The data of 90 puerperae undergoing cesarean section in our hospital from January 2019 to January 2020 were retrospectively analyzed. According to the order of admission, they were equally divided into the control group (CG) and experimental group (EG). Puerperae or their legal guardians had signed the informed consent and volunteered to take part in the study.

### 2.2. Enrollment of Research Subjects

#### 2.2.1. Inclusion Criteria

The inclusion criteria were as follows: puerperae had single pregnancy and in line with cesarean section indications; puerperae had the clinical manifestations such as the amount of bleeding over 500 ml after postpartum 24 h, nausea, and vomiting; puerperae had no taboos or allergic reactions to the drugs used in this study; puerperae were aged over 18 years old with the gestational age over 32 weeks; puerperae had the ASA grade (physical status classified by American Society of Anesthesiologists) [14] as level 2; puerperae had no coagulation dysfunction; and the present study followed the Declaration of Helsinki [15].

#### 2.2.2. Exclusion Criteria

The exclusion criteria were as follows: puerperae with twin or multiple pregnancies; puerperae with blood loss over 400 ml in preoperative assessment, such as placenta implantation; puerperae with hematological and autoimmune diseases; puerperae with prepregnancy hypertension; puerperae with a psychiatric history; puerperae who continued to take anticoagulant drugs before surgery; puerperae with severe anemia before surgery; and puerperae with the gestational hypertension and contraindications to drugs used in this study.

### 2.3. Methods

Both groups of pregnant women underwent cesarean section after epidural anesthesia. After delivery, CG received the intramuscular injection of 5–10 U of oxytocin (manufacturer: Chengdu Hepatunn Pharmaceutical Co., Ltd.; NMPA approval no. H51021982; specification: 1 ml: 5 U) or an intravenous infusion of 5–10 U of oxytocin plus 5% of glucose injection. Additionally, CG also received intravenous infusion of 0.25 g–0.5 g of tranexamic acid injection (manufacturer: Guangzhou Baiyunshan Tianxin Pharmaceutical Co., Ltd.; NMPA approval No. H20056987; specification: 10 ml: 0.5 g), wherein the intravenous infusion was dissolved with 5%–10% of glucose injection.

EG was treated with Baogong Zhixue granules combined with tranexamic acid injection, in which Baogong Zhixue granules (manufacturer: Tianjin Zhongsheng Haitian Pharmaceutical Co., Ltd.; NMPA approval no. Z20103059; specification: 15 g/bag) were administrated with boiled warm water, 1 bag/time, 2 times/day. The usage and dosage of tranexamic acid injection (manufacturer: Guangzhou Baiyunshan Tianxin Pharmaceutical Co., Ltd.; NMPA approval no. H20056987; specification: 10 ml: 0.5 g) were the same as those in CG.

Both groups were treated for 7 days.

### 2.4. Observation Indexes

The amount of bleeding at 2 h and 24 h after delivery was evaluated by the gauze weighing method. The method was as follows. The sterile gauze was weighed preoperatively, and the bloody gauze was weighed again postoperatively to obtain the difference value by subtracting the preoperative weight of sterile gauze, while the blood loss in the aspirator was added to accurately calculate the blood loss during surgery.

Fasting venous blood (3 mL) was collected from both groups, and serum was placed in a centrifuge tube at a 37°C environment to promote its coagulation. After blood was coagulated, the supernatant (serum) was obtained using the centrifugation after equilibrium, and it was carefully sucked out as a standby by the subpackage. An automatic coagulation analyzer (manufacturer: Sysmex Corporation; model: CA-560) was used to detect APTT (activated partial thrombin time) and PT (prothrombin time) with the coagulation method and to detect the Fib (fibrinogen) with the CLUSS method.

The hemodynamics of both groups at 24 h after delivery was monitored, including heart rate (HR) and mean arterial pressure (MAP).

The descending speed of uterine fundus, maintenance time of uterine contraction, and lochia maintenance time of both groups were observed and recorded.

After 5 mL of fasting venous blood was taken from both groups, enzyme-linked immunosorbent assay (ELISA) was adopted to detect the sex hormone indexes such as follicle-stimulating hormone (FSH), luteinizing hormone (LH), and estradiol (*E*_2_).

### 2.5. Statistical Processing

All experimental data were statistically analyzed and processed by the SPSS 21.0 software and graphed by GraphPad Prism 7 (GraphPad Software, San Diego, USA). Enumeration data were tested by *X*^2^ and expressed as (*n* (%)), while measurement data were tested by the *t*-test and expressed as ($\bar{x}$ ± *s*). When *P* < 0.05, the differences were statistically significant.

## 3. Results

### 3.1. Comparison of Baseline Data

No notable differences in gestational age, average age, height, BMI, preoperative coagulation indexes, education, occupation, marriage, and residence were observed between the two groups (*P* > 0.05), as given in Table 1.

### 3.2. Comparison of Postpartum Hemorrhage at Different Time Points

The amount of bleeding at 2 h and 24 h after delivery was less in EG than in CG (*P* < 0.001), as shown in Figure 1.

### 3.3. Comparison of Postpartum Coagulation Indexes

Table 2 provides the remarkably lower APTT and PT and higher Fib after delivery in EG than in CG (*P* < 0.001).

### 3.4. Comparison of Hemodynamic Indexes at 24 h after Delivery

Compared with CG, EG had obviously lower HR and MAP at 24 h after delivery (*P* < 0.001), as shown in Figure 2.

### 3.5. Comparison of Descending Speed of Uterine Fundus, Maintenance Time of Uterine Contraction, and Lochia Maintenance Time

Compared with CG, EG had higher descending speed of uterine fundus, shorter maintenance time of uterine contraction, and shorter postpartum lochia maintenance time (*P* < 0.001), as given in Table 3.

### 3.6. Comparison of Postpartum Sex Hormone Indexes

The postpartum FSH and LH in EG were notably lower than those in CG (*P* < 0.001), with higher *E*_2_ in EG than in CG (*P* < 0.001), as given in Table 4.

## 4. Discussion

Related studies have shown that maternal mortality caused by obstetric hemorrhage ranks first in maternal deaths, and obstetric blood consumption takes third place in the clinical use of blood, accounting for 6% of total blood transfusion volume [16]. Postpartum hemorrhage (PPH), a common complication of cesarean section, is mainly caused by maternal physical weakness, emotional tension, and injuries of the uterine muscle wall, adding to the risk of perioperative maternal deaths if no timely and effective treatment is taken for puerperae. With the continuous development of medicine, drugs for preventing PPH after cesarean section are gradually diversified [17, 18]. Fahrenholtz et al. [19] reported that PPH mostly occurs within 2 hours after delivery and uterine atony bleeding accounts for more than 70%, so uterotonic drugs are mainly used for postpartum treatment in clinic. Oxytocin is a drug frequently used in clinics, but its action time can hardly meet the requirements of persistent uterine contraction. Therefore, other hemostatic drugs should be combined to prevent PPH. Tranexamic acid injection has been proved to be effective in the treatment and prevention of PPH, and its combination with oxytocin has a remarkable effect. However, a few scholars believe that compared with oxytocin treatment, Baogong Zhixue granules combined with tranexamic acid injection can better promote the uterine contraction of patients and accelerate the process of postpartum uterine involution [20]. In this study, the amount of bleeding in EG was notably lower compared with CG at 2 h and 24 h after delivery (*P* < 0.001), suggesting that Baogong Zhixue granules combined with tranexamic acid injection have a more obvious hemostatic effect. The reason is that Baogong Zhixue granules contain various traditional Chinese medicine (TCM) drugs such as Radix Bupleuri and pseudoginseng, whose combination can effectively play the role of cooling blood for hemostasis. In addition, tranexamic acid injection can effectively inhibit the fibrinolytic activity of fibrinolytic enzymes, competitively resist fibrinolytic activators, and inhibit fibrin clot dissolution, thus preventing PPH. APTT is a relatively sensitive test commonly used in clinical screening for the normality of the endogenous coagulation system, which is also an important indicator to reflect the activities of coagulation factors VIII, I, and IX. PT is also an important indicator reflecting the extrinsic coagulation pathways, which can also reflect the activity of patients' own coagulation factors. Fib is a kind of fibrinogen and its abnormal level can lead to coagulation dysfunction. Maternal complications during pregnancy will lead to significantly increased bleeding tendency. The postpartum coagulation indexes APTT, PT, and Fib were better in EG than those in CG, indicating that Baogong Zhixue granules combined with tranexamic acid injection improve the coagulation function of parturient and thus enhance blood microcirculation, which was consistent with the results of Kohn et al. [21].

Dyanna et al. [22] stated in their study that Baogong Zhixue granules combined with tranexamic acid injection have a remarkable hemostatic effect. Van der Nelson et al. [23] showed that Baogong Zhixue granules combined with tranexamic acid injection have a significant clinical effect on treating persistent vaginal bleeding after drug abortion and can effectively stabilize the hemodynamics of patients, with high safety and a certain promotion value in clinics. Besides, Erkan et al. [24] observed that Baogong Zhixue granules combined with tranexamic acid can cause changes in maternal hemodynamics, and the fluctuations of hemodynamics are closely related to maternal prognosis. This study showed that the hemodynamic indexes HR and MAP at 24 h after delivery in EG were remarkably lower compared with CG (*P* < 0.05), demonstrating that Baogong Zhixue granules combined with tranexamic acid injection have little effect on the hemodynamics of pregnant women. In addition, a related report has shown that PPH patients generally experience reproductive system damage due to surgical injury and bleeding, which is very unfavorable for patients with fertility requirements [25]. The clinical research on the PPH treatment after cesarean section shows that PPH can affect the reproductive system in many aspects, among which the uterine involution and sex hormone indexes are common ones. In this study, EG achieved higher descending speed of uterine fundus, shorter maintenance time of uterine contraction and lochia, and better sex hormone indexes compared with CG (*P* < 0.001), fully proving that Baogong Zhixue granules combined with tranexamic acid injection have a positive effect on maternal uterine involution, with little effect on the maternal reproductive system. Due to limited time, this study has some inadequacies, including a small sample size and lack of long-term follow-up. Therefore, it is necessary to expand the sample size, improve the experimental design, and extend the follow-up time in the subsequent research studies to provide a scientific theoretical basis for clinical practice.

In conclusion, Baogong Zhixue granules combined with tranexamic acid injection have a remarkable effect on PPH patients after cesarean section, with little effect on the hemodynamics and reproductive system, which is recommended for clinical treatment.

## Figures and Tables

**Figure 1:** Comparison of postpartum hemorrhage at different time points ($\bar{x}$ ± *s*). (a) Comparison of amount of bleeding at 2 h after delivery. The abscissa represents EG and CG, and the ordinate represents the amount of bleeding at 2 h after delivery (ml). The amount of bleeding at 2 h after delivery was (225.27 ± 25.92) ml in EG and (351.40 ± 35.34) ml in CG. ^*∗*^Difference in the amount of bleeding at 2 h after delivery between the two groups (*t* = 19.306, *P* < 0.001). (b) Comparison of amount of bleeding at 24 h after delivery. The abscissa represents EG and CG, and the ordinate represents the amount of bleeding at 24 h after delivery (ml). The amount of bleeding at 24 h after delivery was (308.38 ± 44.24) ml in EG and (451.20 ± 37.02) ml in CG. ^*∗∗*^Difference in the amount of bleeding at 24 h after delivery between the two groups (*t* = 16.608, *P* < 0.001).

**Figure 2:** Comparison of hemodynamic indexes at 24 h after delivery ($\bar{x}$ ± *s*). (a) Comparison of HR at 24 h after delivery. The abscissa represents EG and CG, and the ordinate represents HR (times/min). The average HR at 24 h after delivery was (83.47 ± 2.99) times/min in EG and (87.20 ± 2.65) times/min in CG. ^*∗*^Difference in HR between the two groups (*t* = 4.584, *P* < 0.001). (b) Comparison of MAP at 24 h after delivery. The abscissa represents EG and CG, and the ordinate represents MAP (mmHg). The average MAP at 24 h after delivery was (77.06 ± 2.05) mmHg in EG and (86.59 ± 3.02) mmHg in CG. ^*∗∗*^Difference in MAP between the two groups (*t* = 17.515, *P* < 0.001).

**Table 1:** Comparison of baseline data.

Items	EG (*n* = 45)	CG (*n* = 45)	*X* ^2^/*t*	*P*
Gestational age (weeks)	33.99 ± 0.62	34.05 ± 0.49	0.509	0.612
Average age ($\bar{x}$ ± *s*, y)	25.18 ± 3.20	25.04 ± 2.62	0.227	0.821
Height (cm)	1.60 ± 0.04	1.61 ± 0.03	1.342	0.183
BMI (kg/m^2^)	20.48 ± 0.26	20.46 ± 0.28	0.351	0.726

Preoperative coagulation indexes				
APTT (S)	43.45 ± 2.00	42.77 ± 2.08	1.581	0.118
PT (S)	18.05 ± 0.62	17.88 ± 0.43	1.511	0.134
Fib (g/L)	2.41 ± 0.06	2.39 ± 0.06	1.581	0.117

Education				
Primary and junior high school	2 (4.44%)	3 (6.67%)	0.212	0.645
High school and college	10 (22.22%)	13 (28.89%)	0.207	0.649
Above college	33 (73.33%)	29 (64.44%)	0.431	0.512

Occupation				
Teachers	4 (8.89%)	5 (11.11%)	0.124	0.725
Company employees	22 (48.89%)	21 (46.67%)	0.045	0.833
Technicians	13 (28.89%)	14 (31.11%)	0.053	0.818
Freelancers	4 (8.89%)	4 (8.89%)	0.000	1.000
Others	2 (4.44%)	1 (2.22%)	0.345	0.557

Marriage			0.104	0.748
Married	40 (88.89%)	39 (86.67%)		
Unmarried	5 (11.11%)	6 (13.33%)		

Residence			0.051	0.822
Urban area	30 (66.67%)	31 (68.89%)		
Rural area	15 (33.33%)	14 (31.11%)		

**Table 2:** Comparison of postpartum coagulation indexes ($\bar{x}$ ± *s*).

Group	*n*	APTT (s)	PT (s)	Fib (g/L)
EG	45	23.36 ± 2.04	10.99 ± 0.28	6.11 ± 0.11
CG	45	32.70 ± 2.78	14.18 ± 0.38	3.96 ± 0.27
*t*		18.170	45.336	49.469
*P*		<0.001	<0.001	<0.001

**Table 3:** Comparison of descending speed of uterine fundus, maintenance time of uterine contraction, and lochia maintenance time ($\bar{x}$ ± *s*).

Group	*n*	Descending speed of uterine fundus (cm/d)	Maintenance time of uterine contraction (d)	Lochia maintenance time (d)
EG	45	1.25 ± 0.11	1.51 ± 0.26	14.70 ± 1.81
CG	45	0.50 ± 0.07	3.00 ± 0.30	18.53 ± 2.47
*t*		38.587	25.178	8.390
*P*		<0.001	<0.001	<0.001

**Table 4:** Comparison of postpartum sex hormone indexes ($\bar{x}$ ± *s*).

Group	*n*	FSH (mU/ml)	LH (mU/ml)	*E*_2_ (pg/ml)
EG	45	6.09 ± 0.25	5.44 ± 0.47	73.40 ± 2.56
CG	45	7.13 ± 0.27	6.92 ± 0.62	66.53 ± 2.60
*t*		18.959	12.761	12.630
*P*		<0.001	<0.001	<0.001

## Data Availability

The data used to support the findings of this study are available from the corresponding author upon request.
